# lncRNA HOTAIR promotes gastric cancer proliferation and metastasis via targeting miR‐126 to active CXCR4 and RhoA signaling pathway

This article has been retracted.

**DOI:** 10.1002/cam4.1302

**Published:** 2019-09-13

**Authors:** Jun Xiao, Hao Lai, Sheng‐Hong Wei, Zai‐Sheng Ye, Fu‐Sheng Gong, Lu‐Chuan Chen

**Affiliations:** ^1^ Department of Gastrointestinal Surgery Fujian Cancer Hospital Fujian Medical University Cancer Hospital Fuzhou 350001 China; ^2^ Department of Gastrointestinal Surgery Guangxi Cancer Hospital Guangxi Medical University Cancer Hospital Nanning 530001 China; ^3^ Department of Molecular immune laboratory Fujian Cancer Hospital Fujian Medical University Cancer Hospital Fuzhou 350001 China

**Keywords:** CXCR4, gastric cancer, HOTAIR, metastasis, miR‐126, RhoA

## Abstract

HOTAIR, a well‐known long noncoding RNAs (lncRNA), has been recognized to contribute to the tumor metastasis in several tumors. But its role in gastric cancer remains elusive. Here, we reported an increase in HOTAIR promoted proliferation and metastasis of gastric cancer cell lines. The HOTAIR and miR‐126 level was determined in 15 paired primary gastric cancer tissues and their adjacent noncancerous gastric tissues. Over‐expression or downregulation HOTAIR was conducted in AGS or BGC‐823 cells to investigate the impact of HOTAIR in proliferation and metastasis. Then dual luciferase reporter assay was utilized to study the interaction between CXCR4 and miR‐126. Cells transfected with shHOTAIR or miR‐126 mimic were subjected to western blot to investigate the role of SDF‐1/CXCR4 signaling in HOTAIR mediated proliferation and metastasis. HOTAIR was highly expressed in gastric cancer tissues and several gastric cancer cell lines. Overexpressed HOTAIR facilitated proliferation and metastasis in vitro while HOTAIR knockdown inhibit proliferation and metastasis. A negative correlation was observed between miR‐126 and HOTAIR. And, we also confirmed the decrease in miR‐126 in clinic specimen. Furthermore, HOTAIR and miR‐126 negatively regulated each other and then increase or decrease CXCR4 expression and downstream pathway, respectively. CXCR4 was confirmed as a direct target of miR‐126. Our study demonstrated that high HOTAIR expression promote proliferation and metastasis in gastric cancer via miR‐126/CXCR4 axis and downstream signaling pathways.

## Introduction

Gastric cancer is the fourth most common cancer and its mortality ranks the second in cancer‐related deaths worldwide 1, 2. Despite that intensive efforts have to be devoted to improving the mortality, patients with advanced or metastatic gastric cancer suffer from widely‐used cytotoxic chemotherapy and poor prognosis 3, 4. Thus, understanding the molecular mechanism of gastric cancer metastasis and its application in novel targeted therapies is urged.

Chemokines are a family of small cytokines or signaling proteins produced by cells 5. They induced chemotaxis in nearby cells, for example, modulating the migration of immune cells by combining with corresponding receptors found on the cell surface 6, 7. Stromal cell‐derived factor ‐1 (SDF‐1), also known as CXCL12, is a ubiquitously expressed chemokine belongs to CXC subfamily of chemokine. It is well‐known as a potent chemoattractant for the homing of hematopoietic stem cells to bone marrow through its canonical receptor CXCR4 8. However, emerging evidences that SDF‐1/CXCR4 plays a critical role in tumor pathogenesis were recognized by recent investigations 9, 10, 11, 12, 13, 14, 15, 16. CXCR4 mRNA level is elevated in the plasma of patients diagnosed with gastric cancer 17. The expression of CXCR4 and SDF‐1 in Intestinal‐type gastric cancer is associated with lymph node and liver metastasis 11. Moreover, the increased CXCR4 in gastric cancer is highly correlated with peritoneal carcinomatosis, accounting for a major cause of mortality in gastric cancer 18. Therefore, it could be a prognostic marker for the overall survival of gastric cancer patients. Carcinoma fibroblasts related SDF‐1/CXCR4 axis recruits endothelial progenitor cells and promotes angiogenesis by increasing vascular endothelial growth factor (VEGF) expression 19, 20. Besides, SDF‐1 was reported to induce proliferation of numerous cancers, including lung cancer, ovarian carcinoma, and pancreatic cancer 21, 22, 23, 24.

Long noncoding RNAs (lncRNAs) are nonprotein‐coding RNA molecules longer than 200 nucleotides. Increasing evidence suggests that dysregulated lncRNAs expression in cancer may be involved in the pathogenesis of cancer and could serve as predictors for outcomes 25. Particularly, lncRNA regulates the translation of messenger RNA (mRNA) by competitively combining with microRNA (miRNA) response element. lncRNA HOX transcript antisense intergenic RNA (HOTAIR), a widely investigated lncRNA, was reported to be upregulated in breast cancer. Enhanced expression of HOTAIR induces genome‐wide re‐targeting of Polycomb repressive complex 2 (PRC2), leading to altered H3 lysine 27 methylation in tumors and increases tumor metastasis in a PRC2‐dependent manner 26.

However, the role and underlying mechanism of HOTAIR in gastric cancer metastasis remains elusive. Here we hypothesize that HOTAIR could mediate proliferation and metastasis through SDF‐1/CXCR4 signaling. Upregulated HOTAIR was observed in both clinical patients with gastric cancer and highly differentiated gastric cancer cell line. We found HOTAIR promoted the proliferation and invasion of gastric cancer cells by regulating miR‐126 expression. More importantly, our study revealed that miR‐126 exert regulatory efficacy through inhibiting downstream SDF‐1/CXCR4 and RhoA signaling.

## Materials and Methods

### Clinical sample

Fifty paired primary gastric cancer tissues and their adjacent noncancerous gastric tissues were collected from Fujian Provincial Tumor Hospital according to standard operation procedures. Patients who had received chemotherapy or radiotherapy were excluded from this study. Resected specimens were immediately frozen in liquid nitrogen and stored at −80°C for the further analysis. The research protocol was designed and approved by the ethical committee of Fujian Provincial Tumor Hospital, and informed consent was obtained from all patients.

### Cell culture

Human gastric mucosal epithelial cell line GES‐1, gastric cancer cell lines SNU‐216, AGS, SGC‐7901 and BGC‐823 cells were obtained from Shanghai Institute of Cell Biology (Shanghai, China) and maintained in PRIM‐1640 (GIBCO, Rockville, MD, USA) with 10% fetal bovine serum (GIBCO), 100 U/mL penicillin, and 100 *μ*g/mL streptomycin in humidified incubator with 5% CO_2_ at 37°C.

### RNA extraction, reverse transcription, and quantitative PCR (qPCR)

Total RNA was extracted with TRIzol reagent (Invitrogen, Carlsbad, CAUSA) according to the manufacturer's instructions and each sample was reversely transcribed to complementary DNA (cDNA) using the PrimeScript^®^ RT reagent Kit with gDNA Eraser (Takara, Dalian, China). Quantitative PCR was employed to determine the relative transcription level of target genes using the SYBR^®^ Premix Ex TaqII kit (Takara). And GAPDH was used as the internal control. The reactions were performed in triplicate for each cDNA on the Applied Biosystems Step One Plus Real‐Time PCR System (Applied Biosystems, Foster city, CA, USA). The relative expressions of HOTAIR and other genes were calculated by 2^−ΔΔct^, according to the widely accepted method. All gene‐specific primers are indicated in Table 1.

**Table 1:** Primers for qPCR

	Forward (5′‐3′)	Reverse (5′‐3′)
HOTAIR	CAGTGGGGAACTCTGACTCG	GTGCCTGGTGCTCTCTTACC
miR‐126	GGCTCGTACCGTGAGTAAT	GTGCAGGGTCCGAGGT
CXCR4	GGAGGGGATCAGTATATACA	GAAGATGATGGAGTAGATGG
RhoA	ATTCGTTGCCTGAGCAATGG	TGTGTCCCACAAAGCCAACT
RhoGEF	GCGCGGACACCAGCC	GCAGACAGCAAAGCAGGG
ARHGAP5	CATCTGTTTTTTGGCCAACCT	GTGGAGGAGCCACAATGTTT
ROCK	ATGTGACTGGTGGTCGGTTG	AACTGGTGCTACAGTGTCTCG
PI3K	TTGTTCCAATCCCAGGTGGA	TTAGCACCCTTTCGGCCTTT
PAK	AGCTGCTACAGGTGAGAAAACT	AGAGGGCATCAGGAGTTGGA
PKN	CATGAGAAGGCTGCTTCGGA	ACTCCTCGTCGAAGTTGCTG
GADPH	ATGTTCGTCATGGGTGTGAA	ATGTTCGTCATGGGTGTGAA

### Plasmids and gene transfection

To construct the HOTAIR expression plasmid, full‐length HOTAIR was amplified by PCR using the primers 5′‐GACTCGCCTGTGCTCTGGAGCT‐3′ and 5′‐TTGAAAATGCATCCAGATTTTT‐3′. Then HOTAIR was cloned into the pcDNA3.1 vector (Invitrogen). The shRNA sequence of the human HOTAIR gene was designed with the BLOCK‐iT^™^ RNAi Designer (Invitrogen). The sequence was chemically synthesized and cloned into pcDNA3.1 vector. Both the miRNA mimic and miRNA inhibitor were synthesized by GenePharma Company (Shanghai, China). Transfection was conducted with Lipofectamine 2000 reagent (Invitrogen, Carlsbad, CA, USA) according to the manufacturer's protocols. After 48 h or 72 h of gene transfection, cells were collected and used for further experiments.

### Cell proliferation assay

Cell proliferation was determined with MTT assay. Cells transfected with indicated plasmid or miRNA were seeded on 96‐well microplates at 1 × 10^4^ cells/well for 48 h. Then medium was removed and 20 *μ*L of MTT assay solution was for 4 h. At the end of the incubation, plates were measured at 570 nm using a microplate reader Model 680 (Bio‐Rad, California, USA). Each experiment has at least three independent tests.

### Crystal violet staining assay

The colony formation of cells was analyzed using a crystal violet staining method. Briefly, cells were trypsinized to single cell suspensions and plated on 6‐well plates and transfected with different genes. After 10‐day incubation in a humidified atmosphere of 5% CO_2_ at 37°C, cells were rinsed with PBS and fixed with 1% glutaraldehyde in PBS overnight in 4°C. Then cells were stained with 0.02% crystal violet in deionized water for 30 min at room temperature. After three water rinses, crystal violet bound to cells was extracted using 70% ethanol at 4°C. Measure the absorbance of each well at 570 nm using a microplate reader Model 680 (Bio‐Rad, California, USA).

### Dual‐luciferase reporter assay

The dual‐luciferase reporter assay was utilized to determine the interaction of miR‐126 and CXCR4 and was conducted according to the method described by Yan et al. 27. Briefly, CXCR4 cDNA fragments containing miR‐126 wild type or mutant binding sites were amplified by PCR and were cloned into the downstream of firefly luciferase gene in pGL3 (Promega, Madison, WI, USA). Then cells in 24‐well plates were co‐transfected with these luciferase reporters and miR‐126 mimic, miR‐126 inhibitor, or corresponding negative controls using Lipofectamine 2000. Forty‐eight hours later, cells were collected and the ratio of firefly luciferase to Renilla luciferase was detected with a Promega Glomax 2020 Single Tube Luminometer instrument (Promega) for each well, where Renilla luciferase intensity worked as internal control. Triplicates were conducted for each experiment.

### Invasion assay

Transwell plates were precoated with Matrigel Matrix (BD Biosciences) and cells were seeded onto matched Transwell membrane inserts. After 48 h incubation in humidified incubator with 5% CO_2_ at 37°C, cells on the lower membrane surface were fixed with 4% paraformaldehyde for 15 min and stained with crystal violet.

### Western blotting

Whole cell extracts were extracted using RIPA and protein concentrations were determined by BCA assay. Equal aliquots of 50 *μ*g total proteins were separated by SDS‐PAGE. Then proteins were transferred to a PVDF membrane. Membranes were blocked with 5% bovine serum albumin in TBST and then incubated in primary antibodies overnight at 4°C followed by secondary antibodies for 1 h at 37°C. Rabbit polyclonal primary antibody against CXCR4 (sc‐9046), mouse monoclonal antibodies against RhoA (sc‐418), RhoGEF (sc‐166301), ROCK (sc‐17794), PI3K (sc‐166365), PAK (sc‐166174), PKN (sc‐136037), GAPDH (sc‐166545), and the horseradish peroxidase‐conjugated secondary antibodies against rabbit‐IgG (sc‐2004) and mouse‐IgG (sc‐2005) were purchased from Santa Cruz Biotechnology. The primary rabbit polyclonal antibody against ARHGAP5 was purchased from Sigma‐Aldrich. Finally, signal was visualized through a chemiluminescent detection system (Pierce ECL Substrate Western blot detection system, Thermo, Rockford, IL, USA).

### Statistical analysis

Data were presented as mean ± SEM. For comparisons between two groups, Student's *t*‐test was employed. The correlation significance was determined by Spearman and Pearson correlation analyses. A two side value of *P* < 0.05 was considered statistically significant. All statistical analyses were performed by GraphPad Prim 5 (GraphPad Software, La Jolla, CA, USA).

## Results

### HOTAIR expression was elevated in gastric cancer tissues and gastric cancer cell lines

Firstly, we collected 15 pairs of cancer tissues and corresponding adjacent noncancer tissues from patients diagnosed as gastric cancer. We found that HOTAIR mRNA was significantly upregulated in cancer sites compared with the normal (Fig. 1A). Then we confirmed the expression level of HOTAIR with five gastric‐originated cell lines. In human normal gastric epithelia cell line GES‐1 and SNU‐216, HOTAIR expression was kept in a relatively low base level (Fig. 1B). In AGS cells, HOTAIR expression was higher than GES‐1. But the difference showed no statistical significance, whereas qPCR demonstrated a dramatic elevation of HOTAIR enrichment in SGC‐7901 cells and BGC‐823 cells than GES‐1 cells.

**Figure 1:** HOTAIR expression elevated in gastric cancer cell lines and gastric cancer tissues. (A) Levels of HOTAIR mRNA were assayed using qRT‐PCR in gastric cancer and the paired normal tissues. (B) Quantified mRNA level in normal or gastric cancer cell lines. Data are means ± SEM.*P < 0.05, **P < 0.01.

### HOTAIR promoted the proliferation and metastasis in gastric cancer cell lines

To identify the effect of upregulated HOTAIR in the gastric cancer, AGS cells, which has low expression of HOTAIR, was transfected with HOTAIR cDNA plasmid (pc‐HOTAIR) or empty vector (pc‐control). qPCR validated that HOTAIR expression was dramatically increased in the pc‐HOTAIR group (Fig. 2A). Two days after HOTAIR overexpression, the cell viability was higher than pc‐control and the difference between two groups was statistic significant at the 4th day (Fig. 2B). Cells in 6‐well plates were stained with crystal violet and foci counted 10 days after transfection, as described in Materials and Methods. Abundant foci were observed in HOTAIR overexpressed AGS cells compared to the pc‐control (Fig. 2C). To investigate the effect of HOTAIR on the invasion of AGS cells, cells migrated through transwell membrane were stained with crystal violet. Microscopic observation revealed an increase in cell number in HOTAIR overexpression group (Fig. 2D).

**Figure 2:** Overexpressed HOTAIR facilitated proliferation and metastasis in AGS. (A) qRT‐PCR. AGS cells were transfected with plasmid of HOTAIR cDNA (pc‐HOTAIR) or control plasmid (pc‐control) and then subjected to qRT‐PCR analysis of HOTAIR levels. (B) Cell viability CCK‐8 assay. AGS cells transfected with pc‐HOTAIR or pc‐control were collected at various days and then subjected to CCK‐8 assay. (C) Colony formation assay. Cells were subjected to colony formation assay. (D) Invasion assay. Cells were subjected to invasion assay and stained with crystal violet. The graph is summarized data of the invasion assay. Data are means ± SEM.*P < 0.05, **P < 0.01.

To further validate the role of HOTAIR in proliferation and metastasis, we downregulated the high expression of HOTAIR in BGC‐823 cells with its specific shRNA (Fig. 3A). As shown in Figure 3B, HOTAIR knockdown significantly inhibited the proliferation of BGC‐823 cells (Fig. 3B). Moreover, the colony formation and invasion capacity were both impaired (Fig. 3C and D). Taken together, these data demonstrated that HOTAIR facilitated the proliferation and migration of gastric cancer cells.

**Figure 3:** Down‐regulated HOTAIR inhibited proliferation and metastasis in BGC‐823 cells. (A) qRT‐PCR. BGC‐823 cells were transfected with plasmid of HOTAIR shRNA (shHOTAIR) or control shRNA (shNC) and then subjected to qRT‐PCR analysis of HOTAIR levels. (B) Cell viability CCK‐8 assay. BGC‐823 cells transfected with shHOTAIR or shNC were collected at various days and then subjected to CCK‐8 assay. (C) Colony formation assay. Cells were subjected to colony formation assay. (D) Invasion assay. Cells were subjected to invasion assay and stained with crystal violet. The graph is summarized data of the invasion assay. Data are means ± SEM.*P < 0.05.

### HOTAIR and miR‐126 had negative correlation in gastric tissue and cancer cell lines

Previous studies demonstrated that HOTAIR could negatively regulate miR‐126 28. To explore whether similar modulatory mechanism was employed by HOTAIR in its regulation of proliferation and metastasis, we firstly checked the miR‐126 level in five gastric‐originated cell lines (Fig. 4A). We observed that normal gastric cells GES‐1 expressed the highest miR‐126, which was dramatically decreased in gastric cancer lines with an opposite expression pattern to that of HOTAIR. Furthermore, miR‐126 level in the same gastric cancer tissues and adjacent noncancer tissues from 15 patients were measured with qPCR. Compared with normal tissues, the expression level of miR‐126 was dramatically reduced in gastric carcinoma tissues (Fig. 4B). More importantly, the correlation line showed that the HOTAIR expression was negatively correlated with that of miR‐126 (Fig. 4C). These data indicated that miR‐126 may participant in the efficacy of HOTAIR in gastric cancer.

**Figure 4:** HOTAIR expression negatively correlated with miR‐126. (A) Quantified mRNA level in normal or tumor gastric cell lines. Data are means ± SEM.*P < 0.05, **P < 0.01. (B) qRT‐PCR. Levels of miRNA were assayed using qRT‐PCR in gastric cancer and the paired normal tissues. (C) The Spearman correlation analysis of miR‐126 and HOTAIR (D) qRT‐PCR. BGC‐823 cells were transfected with shHOTAIR or shNC and then subjected to qRT‐PCR analysis of miR‐126 levels. (E) qRT‐PCR. BGC‐823 cells were transfected with plasmid of miR‐126 mimics (mimic NC) or miR‐126 mimics or plasmid of miR‐126 inhibitor (inhibitor NC) or miR‐126 inhibitor, and then subjected to qRT‐PCR analysis of miR‐126 levels. (F) qRT‐PCR. BGC‐823 cells were transfected with plasmid of mimic NC or miR‐126 mimics or inhibitor NC or miR‐126 inhibitor and then subjected to qRT‐PCR analysis of HOTAIR levels. (G) qRT‐PCR. AGS cells were transfected with pc‐control or pc‐HOTAIR and then subjected to qRT‐PCR analysis of miR‐126 levels. (H) qRT‐PCR. AGS cells were transfected with plasmid of mimic NC or miR‐126 mimics or inhibitor NC or miR‐126 inhibitor, and then subjected to qRT‐PCR analysis of miR‐126 levels. (I) qRT‐PCR. AGS cells were transfected with plasmid of mimic NC or miR‐126 mimics or inhibitor NC or miR‐126 inhibitor and then subjected to qRT‐PCR analysis of HOTAIR levels. Data are means ± SEM.*P < 0.05, **P < 0.01.

We used pc‐DNA and shRNA to upregulate or downregulate HOTAIR in AGS and BGC‐823 respectively. In HOTAIR overexpressed AGS cells, miR‐126 obviously decreased compared to the pc‐control, whereas silence expression of HOTAIR in BGC‐823 cells elevated miR‐126 level (Fig. 4D and G). miR‐126 mimic or miR‐126 inhibitor was transfected into BGC‐823 cells and AGS cells, transfection efficiency was validated by qPCR (Fig. 4E and H), and we observed similar negative correlation between HOTAIR and miR‐126. The expression of HOTAIR in BGC‐823 cells and AGS cells transfected with miR‐124 mimics was decreased while miR‐124 inhibitor elevated HOTAIR level (Fig. 4F and I).

### miR‐126 inhibited the proliferation and metastasis in gastric cancer cells

According to the negative correlation between miR‐126 and HOTAIR, investigation the effect of miR‐126 on gastric cancer was conducted. miR‐126 mimic was utilized to validate the effect of miR‐126 in gastric cancer. The proliferation in miR‐126 mimic group was dramatically decreased after miR‐126 mimic transfection for 4 days compared to the mimic NC group in BGC‐823 cells (Fig. 5A). Meanwhile, the colony number also dropped and fewer cells were observed to transmigrate through the transwell membrane in the invasion assay (Fig. 5B and C). Furthermore, we silenced miR‐126 in AGS cells. Cells transfected with miR‐126 inhibitor exhibited opposite trends with elevated cell viability, colony formation, and enhanced transmigration capability (Fig. 5D–F). Thus, we verified that miR‐126 inhibit the proliferation and migration in gastric cancer.

**Figure 5:** Overexpressed miR‐126 inhibits proliferation and metastasis of gastric cancer cells. (A) Cell viability CCK‐8 assay. BGC‐823 cells transfected with miR‐126 mimics or control plasmid (mimic NC) were collected at various days and then subjected to CCK‐8 assay. (B) Colony formation assay. BGC‐823 cells were subjected to colony formation assay. (C) Invasion assay. BGC‐823 cells were subjected to invasion assay and stained with crystal violet. The graph is summarized data of the invasion assay. (D) Cell viability CCK‐8 assay. AGS cells transfected with miR‐126 inhibitor or control plasmid (mimic NC) were collected at various days and then subjected to CCK‐8 assay. (E) Colony formation assay. AGS cells were subjected to colony formation assay. (F) Invasion assay. AGS cells were subjected to invasion assay and stained with crystal violet. The graph is summarized data of the invasion assay. Data are means ± SEM.*P < 0.05.

### HOTAIR and miR‐126 regulated the proliferation and metastasis in gastric cell lines via CXCR4 pathways

Previous studies reported the tumor suppressor role of miR‐126 in colon cancer by negatively regulating SDF‐1/CXCR4 and RhoA signaling 29, 30, 31.Thus, we examined downstream proteins of both pathways in gastric cancer cells. Real‐time PCR results observed a significant increase in CXCR4 and RhoGEF, a critical protein in RhoA activation, and downregulation of ARHGAP5 at the mRNA level in HOTAIR knockdownedBGC‐823 cells (Fig. 6A). Similar, miR‐126 mimic transfection dramatically decreased the mRNA of RhoA, RhoGEF, and downstream ROCK while elevated ARHGAP5 mRNA (Fig. 6B). Western blot validated that CXCR4, RhoGEF, ROCK, PI3K, PAK, and PKN expression was reduced in miR‐126 overexpression BGC‐823 cells; whereas ARHGAP5 was upregulated (Fig. 6C). Meanwhile, the expression profile of cells overexpressing HOTAIR was opposite, with increased CXCR4, RhoGEF, PI3K, ROCK, PAK, and PKN and downregulated ARHGAP5. To further confirm the results in BGC‐823 cells, AGS cells were also utilized to investigate the expression change in miR‐126/CXCR4 signaling after HOTAIR overexpression transfection or miR‐126 knockdown. The results were consistent with that in BGC‐823 cells as HOTAIR overexpression activate or miR‐126 knockdown activated or inhibited CXCR4/RhoA signaling, respectively (Fig. 6D–F).

**Figure 6:** HOTAIR promotes the proliferation and metastasis in gastric cell lines via miR‐126/CXCR4/RhoA pathways. (A) qRT‐PCR. BGC‐823 cells were transfected with plasmid of HOTAIR shRNA (sh‐HOTAIR) or control plasmid (shNC) and then subjected to qRT‐PCR analysis of indicated mRNA levels. (B) qRT‐PCR. BGC‐823 cells were transfected miR‐126 mimics or control plasmid (mimic NC) and then subjected to qRT‐PCR analysis of indicated mRNA levels. (C) Western blot. BGC‐823 cells were transfected with shNC, or sh‐HOTAIR, or mimic NC, or miR‐126 mimics for 48 h and then subjected to western blot analysis of protein expression. (D) qRT‐PCR. AGS cells were transfected with plasmid of pc‐control or pc‐HOTAIR and then subjected to qRT‐PCR analysis of indicated mRNA levels. (E) qRT‐PCR. AGS cells were transfected with miR‐126 inhibitor or plasmid of miR‐126 inhibitor (inhibitor NC) and then subjected to qRT‐PCR analysis of indicated mRNA levels. (F) Western blot. AGS cells were transfected with pc‐control or pc‐HOTAIR, or inhibitor NC, or miR‐126 inhibitor for 48 h and then subjected to Western blot analysis of protein expression. (G) Illustration of CXCR4 mutation plasmids for luciferase reporter assay. CXCR4 mutation locates at 239–245 of the miR‐126 3′‐UTR. (H) Luciferase reporter assay. BGC‐823 cells were co‐transfected with CXCR4‐3′ UTR wide type or CXCR4‐3′ UTR mutation plasmids together with miR‐126 mimic or mimic NC and then subjected to the luciferase assay. Data are means ± SEM. *P < 0.05, **P < 0.01.

Furthermore, CXCR4 mutation was applied to validate the interaction between CXCR4 and miR‐126. It was reported that CXCR4 mRNA 3′‐UTR contained a miR‐126 matched site at position 239–245 32. Thus, we transfected BGC‐823 cells with miR‐126 mimic or NC mimic and luciferase report plasmid with CXCR4 wild type 3′UTR or mutant 3'UTR, which contains two mutated sites at predicted binding position 239–245 (Fig. 6G). Luciferase assay demonstrated that miR‐126 downregulated luciferase activities controlled by wild type CXCR4 3′UTR but did not affect luciferase activities transfected with mutant CXCR4 3′UTR (Figs. 6H, 7).

Therefore, our data revealed that lncRNA HOTAIR and miR‐126 modulated proliferation and invasion through CXCR4 and the downstream RhoA signaling pathway in gastric cancer cell lines.

## Discussion

lncRNAs are a class of noncoding RNA with over 200 nt in length and usually have complex and diverse sequences. In mammals, lncRNAs comprise over 50% of the total number of RNAs transcribed by RNA polymerase II. Emerging evidences demonstrated that lncRNA are novel master regulators of tumorigenesis, progression and therapy response in various human diseases including cancer 25.

HOTAIR, a 2.2 kb long transcript with six axons, was firstly identified in the nucleus of breast cancer cells, especially metastasized breast cancers. HOTAIR is coexpressed with HOXC gene cluster and could regulate various genes 33. For example, HOTAIR could bind to PRC2 complex and alter H3K27 methylation and gene expression to induce tumor cell invasiveness and metastasis 26. During epithelial‐mesenchymal transition (EMT), HOTAIR could repress the expression of WIF‐1, an inhibitor of Wnt/*β*‐catenin pathway that mediates EMT in esophageal cancer cells 34. Present study showed that HOTAIR was upregulated in gastric cancer tissue and cell lines and demonstrated that HOTAIR overexpression is associated with proliferation and migration in gastric cancer, which is consistent with investigations from previous reports 27.

MicroRNAs (miRNAs) are endogenous noncoding RNAs with a length around 21–23 nt. MiRNAs function by binding to Argonaute (Ago) protein and constitute RNA induced silencing complex (RISC), a ribonucleoprotein complex 35. This complex could be tethered to complementary mRNAs, resulting in mRNA degradation. Nowadays, miRNAs have become firmly identified as key regulators of cancer 36. In this study, we focus on miR‐126, which has been shown to be frequently downregulated in a variety of malignancies and act as a potential tumor suppressor 37. miR‐126 has been validated to be downregulated in gastric cancer and upregulation of miR‐126 might suppress the malignant phenotypes of gastric cancer cells via targeting oncogene Crk and PI3KR2 38, 39. Our study found that the suppression of miR‐126 in gastric cancer tissue and cell lines and overexpression of miR‐126 did suppress the colony formation and migration of BGC‐823 cells, which consist with previous studies.

lncRNA and miRNA negatively regulated each other in many cancer types. It is reported that in osteosarcoma cells, HOTAIR knockdown could upregulated miR‐126 and then inhibited DNMT1 to regulate DNA methylation, which indicated a negative correlation between HOTAIR and miR‐126 28. In this study, we found that HOTAIR knockdown mimic the inhibition of proliferation and metastasis from miR‐126 overexpression and mutual negative regulation between HOTAIR and miR‐126 is validated in gastric cancer tissue and cell lines. However, the underlying mechanism by which HOTAIR regulates miR‐126‐3p (miR‐126 utilized in this study) remains elusive. In previous study, Yan et al. validated that miRNAs, selected miR‐126‐5p, are direct targets of HOTAIR with online software Diana Tool 40 while the sequence prediction tool did not reveal predictive bonding site between HOTAIR and miR‐126‐3p (data not shown). Li et al. found that HOTAIR could repress the expression of CDKN2A through inhibiting the promoter activity of CDKN2A by DNA hypermethylation 28. Thus, we hypothesized that HOTAIR might similarly negatively regulate miR‐126 in an indirect manner, such as upstream transcription factor regulation. Further investigation will be conducted in our future study to clarify the detailed mechanism.

Reports have showed that miR‐126 functioned as a metastasis suppresser in thyroid cancer and colorectal cancer cells via targeting CXCR4 30, 32. Present study showed that miR‐126 exert similar anti‐metastasis effect via directly targeting CXCR4 3′UTR in gastric cancer. Chemokines, small proinflammatory chemoattractant cytokines that bind to specific GPCR, could be divided into four groups according to the number and position of conserved cysteines, named CXC, CC, C and CX3C. SDF‐1 is a widely expressed CXC chemokine and functions through its canonical receptor CXCR4. The SDF‐1/CXCR4 overexpression in tumor cells lead to autocrine/paracrine stimulation of cancer cells, increasing tumor metastasis 41. In gastric cancer, SDF‐1 activated CXCR4 could upregulated the expression of MMP‐2 and MMP7, which plays an important role in the degradation of the extracellular matrix 42. Therefore, in next section, we tested whether HOTAIR may facilitate metastasis in gastric cancer via miR‐126/CXCR4 axis. The results validated that HOTAIR and mir‐126 could respectively active or inhibit CXCR4 and the signaling pathways downstream, including RhoA/Rock and PI3K pathway. This result is supported by Wei Yuan's study which demonstrated that miR‐126 could inhibit CXCR4/RhoA pathway in colon cancer. 29. Another study indicated a consistence between RhoA expression and the results of a functional study on miR‐126. In particular, miR‐126 downregulated Rho/Rac guanine nucleotide exchange factor 2 and elevated Rho GTPase‐activating protein 5, followed by inactivation of Rho GTPase and the Rho GTPase signaling pathway, to exert its tumor suppressor role in colon cancer cells 43. This study suggested that HOTAIR/miR‐126 may also regulate RhoA signaling via direct interaction. Further mechanism should be validated in future study.

In conclusion, our study identified the critical role of lncRNA HOTAIR/miR‐126/CXCR4/RhoA axis as in gastric cancer, providing a new thought for the targeted therapy of gastric cancer.

## Conflict of Interest

None.
